# Identification and characterization of genes related to salt stress tolerance within segregation distortion regions of genetic map in F_2_ population of upland cotton

This article has been retracted.

**DOI:** 10.1371/journal.pone.0247593

**Published:** 2021-03-26

**Authors:** Muhammad Shehzad, Zhongli Zhou, Allah Ditta, Majid Khan, Xiaoyan Cai, Yanchao Xu, Amir Maqbool, Ahlam Khalofah, Muhammad Shaban, Muhammad Naeem, Mohammad Javed Ansari, Kunbo Wang, Fang Liu

**Affiliations:** 1 State Key Laboratory of Cotton Biology, Institute of Cotton Research, Chinese Academy of Agricultural Sciences, Anyang, Henan, P.R China; 2 Plant Breeding, and Genetics Division, Cotton Group, Nuclear Institute for Agriculture and Biology (NIAB), Faisalabad, Punjab, Pakistan; 3 Department of Agricultural Genetic Engineering, Faculty of Agricultural Sciences and Technologies, Nigde Omer Halisdemir University, Nigde, Turkey; 4 Biology Department, Faculty of Science, King Khalid University, Abha, Saudi Arabia; 5 Department of Plant Breeding and Genetics, Faculty of Agricultural Science & Technology, Bahauddin Zakariya University, Multan, Pakistan; 6 Department of Botany, Hindu College Moradabad (Mahatma Jyotiba Phule Rohilkhand University Bareilly), Bareilly, India; 7 School of Agricultural Sciences, Zhengzhou University, Zhengzhou, Henan, China; Harran Üniversitesi: Harran Universitesi, TURKEY

## Abstract

Segregation distortion (SD) is a genetic mechanism commonly found in segregating or stable populations. The principle behind this puzzles many researchers. The F_2_ generation developed from wild *Gossypium darwinii* and *G*. *hirsutum* CCRI12 species was used to investigate the possible transcription factors within the segregation distortion regions (SDRs). The 384 out of 2763 markers were distorted in 29 SDRs on 18 chromosomes. Good collinearity was observed among genetic and physical maps of *G*. *hirsutum* and *G*. *barbadense* syntenic blocks. Total 568 genes were identified from SDRs of 18 chromosomes. Out of these genes, 128 belonged to three top-ranked salt-tolerant gene families. The DUF597 contained 8 uncharacterized genes linked to Pkinase (PF00069) gene family in the phylogenetic tree, while 15 uncharacterized genes clustered with the zinc finger gene family. Two hundred thirty four miRNAs targeted numerous genes, including ghr-miR156, ghr-miR399 and ghr-miR482, while others targeted top-ranked stress-responsive transcription factors. Moreover, these genes were involved in the regulation of numerous stress-responsive cis-regulatory elements. The RNA sequence data of fifteen upregulated genes were verified through the RT-qPCR. The expression profiles of two highly upregulated genes (*Gh_D01G2015* and *Gh_A01G1773*) in salt-tolerant *G*. *darwinii* showed antagonistic expression in *G*. *hirsutum*. The results indicated that salt-tolerant genes have been possibly transferred from the wild *G*. *darwinii* species. A detailed functional analysis of these genes can be carried out which might be helpful in the future for gene cloning, transformation, gene editing and the development of salt-resistant cotton varieties.

## Introduction

Segregation distortion (SD) is deviation of the observed allelic frequencies at a locus from expected Mendelian ratio, of a given genotypic class in a segregating population. In the construction of a genetic map, some chromosomal regions exhibit segregating alleles by deviating their anticipated Mendelian ratios towards a particular allele. These alleles tend to cluster at small genomic regions within a chromosome, known as segregation distortion regions (SDRs). Distorted markers bring errors leading to disturbance in the orders of genetic markers and influence the calculation of genetic distance [1]. Accordingly, it affects the genetic mapping of morphological characteristics [2]. This phenomenon is widespread in both plants and animals [3]. The SD phenomenon is not extensively studied in crops; however, markers with segregating ratios have been described in most of the crops, including maize [4], barley [5], potato [6], wheat [7], rapeseed [8] and cotton [9]. The 14 SDRs were found on nine chromosomes in maize and four of these were closely linked to gametophyte genes, proposing the evolution of SDRs [10]. Lu et al. [3] identified 18 SDRs on 10 chromosomes of maize and 3 gametophytic genes were potentially acting as genetic prompts of SDRs [3]. The 14 SDRs were reported from barley and their association was compared between known SDRs and haploid genes [11]. Similarly, a higher number of distortions have been reported in *Medicago sativa* L., with 24% of distortions found in F_1_ mapping generation and 34% in F_2_ mapping generation, resulting high distortion level per linkage [12, 13]. Correspondingly, SDRs in double haploid rice recombinant inbred has been detected on 9^th^ chromosome [4].

Several mechanisms can cause SD and male gametes have major SD in most of the organisms [14]. Similarly, in cotton, most of the SDs were primarily skewed from the male instead of the female population on some of the chromosomes [15]. Previously, several studies have been directed towards unraveling SDRs in cultivated cotton, but little research has been carried out on discovering these in F_2_ population developed from wild cotton paternal species. Furthermore, insufficient research has concentrated on the determination of important genes harbored within SDRs [16]. Most recent effort in this regard has been done to develop a BC_2_F_2_ population between *Gossypium hirsutum* and *G*. *mustelinum* exploring the SDRs in wild cotton progenitors [16]. In an earlier study, we developed a F_2_ population of 188 individuals to generate a highly dense genetic map of 2763 polymorphic markers on all 26 chromosomes [17]. A total 384 markers were distorted on 18 chromosomes, harboring the highest number of SDRs. So far, little information is available about the genetic phenomena of SDs in cotton. In this study, we analyzed SDRs in a previously constructed genetic map of *G*. *hirsutum* and *G*. *darwinii*, a wild species of cotton. Wild *G*. *darwinii* species originated from Galapagos Island and had a similar genetic architecture to *G*. *barbadense*. It is characterized by the presence of valuable traits like abiotic stress tolerance, fiber fineness and resistance against *Verticillium* and *Fusarium* wilts [17]. *G*. *hirsutum* is predominantly grown variety in the world [18]. Genetic diversity of different crop species, including wheat, rice and cotton have been improved by using their wild progenitors [19].

Salt stress is threatening the production of many crops globally. It affects cotton productivity around the world. An excess of carbonates, bicarbonates and chlorides of calcium, magnesium, and sodium in the soil leads to soil salinization. The reduction in crop production due to salt and drought stress, and heavy metal pollution is estimated to be >50% compared with other stresses [20]. Globally, 954.8 million ha of cultivated land are affected by salts [21]. Every year, there is 10% increase in salinized areas worldwide [22]. The NaCl is the most prevalent salt in the soil predominantly in the form of cations (Na^+^) and anions (Cl^-^) that affects nutrition and causes ion imbalance. An excess of Na^+^ ions interferes with the concentration of Ca^2+^ and Mg^2+^ ion within the soil leading to osmotic changes. It ultimately affects critical biochemical processes that result in stunted growth [23].

The plants possess various homeostasis protection mechanisms to mitigate harmful effects of stress. Calcium is a common second messenger playing a vital role in plant development under different biotic and abiotic stresses. When plants are exposed to salt stress, temporary variations in the concentration of calcium are produced in the cytoplasm. These variations are detected and decoded by a specific set of calcium sensors, including calmodulins (CaM), calmodulin proteins (CaML), calcineurin B proteins (CBL) and calcium-dependent protein kinases (CDPK). It has been previously shown that Pkinase changes the reactions of plants to osmotic and salt stress. Similarly, zinc finger family is actively involved in the recognition and packaging of DNA and RNA, transcriptional regulation, apoptosis, assembly, folding of proteins and lipid binding [24]. Interestingly, MYB family genes predominantly occur in plants similarly to other animals and fungi, playing a key role in abiotic stress, plant development, signal transduction and resistance against diseases [25, 26].

Upland cotton is economically important crop and main source of natural fiber for textile mills. Its fiber quality and yield are severely affected by different stresses [27]. Cotton crop is adversely affected by salinity stress in different ways such as lower seed germination and stunted vegetative growth leading to lower crop yield and fiber output. In this study, we analyzed SDRs from a genetic map created from allotetraploid and diploid cotton in the D genome using simple sequence repeat (SSR) markers. We particularly focused on the chromosomes that showed SDs of markers during the construction of the genetic map. We subsequently mined the SDRs for the presence of vital genes and used the genetic map to discover some of the important gene families having major effect on plant development in relation to salt stress. Consequently, 105 genes of top 3 salt stress-tolerant families and 23 uncharacterized genes were noted in SDRs of *G*. *hirsutum*, *G*. *arboreum* and *G*. *raimondii*. Furthermore, recognized genes were subjected to detailed investigation such as phylogenetic analysis, gene structure, subcellular localization, possible gene ontology-based functions, miRNAs, cis-elements, and expression profile in leaves and roots of *G*. *darwinii* and *G*. *hirsutum* under salt stress.

## Materials and methods

### Parent resources

In the current study, F_2_ multiple lines were used and established by crossing *G*. *hirsutum* CCRI12 and *G*. *Darwinii* 07. The *G*. *hirsutum* CCRI12 was developed by the Institute of Cotton Research, Chinese Academy of Agricultural Sciences (CAAS), Anyang, Henan Province, China. This variety is high yielding but prone to numerous abiotic stresses [28]. Wild *G*. *darwinii* species has originated from Galapagos Island (imported and maintained by Institute of Cotton Research, Chinese Academy of Agricultural Sciences Anyang, Henan Province, China) and closely related to *G*. *barbadense* in terms of fiber fineness, salt and drought tolerance along with resistance to *Verticillium* disease [17]. JoinMap software was used for the development of genetic map [29]. The F_2_ segregating population was used for the construction of this genetic map, mainly composed of EST-SSR primers accessible at Cotton Marker Database (CMD), including ESTs-SSRs and gSSRs markers, http://www.cottonmarker.org [17]. The 384 polymorphic markers within SDRs were used in this study. These 384 markers were found in 29 SDR regions out of 2763 located on 18 chromosomes. The physical positions of 214 markers were downloaded from cotton functional genomics database (cottonFGD) website (https://cottonfgd.org). The genetic and physical positions of these markers were used in CIRCOS v0.69 (Circular Genome Data Visualization) for collinearity analysis [30].

### Identification of genes from SSR Markers

All identified gene sequences from SDR markers were downloaded from cotton functional genomic database (https://cottonfgd.org) in NAU (Nanjing Agriculture University) assembly. The BLASTx with E-value 1×10^−5^ and identity >80% was used to find genes in the genomes of *G*. *hirsutum*, *G*. *arboreum* and *G*. *raimondii*. Previously, these methods have been employed by Ditta et al. [31]. Meanwhile, the identified candidate genes from SSR markers found within SDRs had already been used by Kirungu et al. [16]. The protein kinase, zinc finger and MYB domain of each gene were confirmed from SMART and PFAM databases (http://smart.embl-heidelberg.de/; http://pfam.xfam.org).

### Phylogenetic analysis

Gene sequences of *G*. *hirsutum*, *G*. *arboreum* and *G*. *raimondii* were aligned using clustal W program [32]. Afterwards, the evolutionary distance was inferred by using neighbor-joining (NJ) method, and a phylogenetic tree was built through molecular evolutionary genetic analysis (MEGA v6.06), based on gene sequences by selecting 1,000 numbers of bootstrap replications. The 8 uncharacterized genes of PLATZ (PF04640), 15 genes belonging to protein of unknown function DUF597 and 23 unidentified genes were designated for function identification and phylogenetic analysis.

### Structural analysis and subcellular localization

Subcellular localization of the three cotton gene families and uncharacterized genes were illustrated by TargetP1.1 server (http://www.cbs.dtu.dk/services/TargetP/) and confirmed the subcellular compartmentalization of all promising genes by WoLFPSORT (https://wolfpsort.hgc.jp/) [33]. The structures of genes was graphically visualized by using Gene Structure Display Server (GSDS 2.0) online software (http://gsds.cbi.pku.edu.cn).

### miRNA and cis-elements analysis

The CDS sequences of *G*. *hirsutum* genes were downloaded from www.cottonfgd.com.org and used for prediction of miRNA, later CDS sequences were blasted in online software, http://bioinformatics.cau.edu.cn/PMRD to obtain miRNA short sequences. Identification of genes that targeted miRNA by both sequences and CDS of genes were applied in an online database psRNATarget server (http://plantgrn.noble.org/psRNATarget/?Function=3). Additionally, genomic DNA sequences in fasta format were downloaded from www.cottonfgd.com.org (cottonFGD) for cis-element analysis. The fasta sequences were submitted in an online plantCARE database (http://bioinformatics.psb.ugent.be/webtools/plantcare/html/) to obtain the cis-elements of the genes.

### Gene ontology

The genes were classified according to their functions into three categories, including molecular functions, cellular component and biological processes. Genetic characteristics and protein features were determined using cotton functional genomic database (cottonFGD) (https://cottonfgd.org). *G*. *hirsutum* was used as the reference genome [39]. The heat map was developed from an expression data of RT-qPCR and RNA sequence, using R statistical package (CSIRO, Mathematical and Information Sciences, Cleveland, Australia ver. 3.4.4).

### Syntenic analysis and duplication of genes

The distribution of genes in the genomes of three cotton species were mapped with Circular Genome Data Visualization (CIRCOS) (version 0.69) programs [30]. The genes distribution on chromosomes was investigated based on the start and end positions. The orthologous genes of *G*. *hirsutum*, *G*. *arboreum* and *G*. *raimondii* were identified by BLASTp with >80% similarity ratio and a minimum 80% alignment ratio according to the length of protein. All homologous genes sequences were aligned with clustalW program in MEGA (v6.06). After alignment, the resulted file from MEGA (6.06) software was given to DNA Sequence Polymorphism (DNaSP) (v. 5.10) to calculate non-synonymous substitution’s site (Ks), synonymous substitution’s site (Ka) and synonymous/nonsynonymous substitution’s site (Ka/Ks) [34]. The MCScanX package was used to determine the duplication of genes [35]. All genes and markers were mapped on the chromosomes of *G*. *hirsutum*, *G*. *arboreum* and *raimondii* by map chart software [36].

### Hydroponic system

In this study, we used hydroponics for salt tolerance instead of saline field as hydroponics provide a uniform salt concentration for all the plants; therefore, ensuring that genes obtained are associated with the salt treatment. An experiment was conducted in greenhouse at the Institute of Cotton Research, Chinese Academy of Agricultural Sciences (CAAS) Anyang, Henan province, China. Three leaf stage seedlings of *G*. *hirsutum* CCRI12 and *G*. *Darwinii* 07 were grown in 200 mM sodium chloride (NaCl) solution in a hydroponic system. The hydroponic system was first described by Oluoch et al. [37], per three replications. Seeds of *G*. *hirsutum* CCRI12 and *G*. *darwinii*07 were surface sterilized in 0.5% sodium hypochlorite (NaOCl) for five min and washed three times with distilled water. Healthy seeds were sorted out after seed grading and germinated in sterile double-layered vertical columned Whatman filter paper in an incubator. The filter papers were soaked in 100 ml of distilled water and placed in the incubator at 32 °C for 3 days. Three parallel seedlings were chosen and transferred to holes of thermo-pore sheets and fixed in the tray with the help of a soft sponge. About seven liters of half-strength modified Hoagland nutrient solution was maintained in every container [38]. Air pumps were attached to each container for aeration in the solution to ensure proper root growth. Temperature in the greenhouse was kept between 27–30 °C with a photoperiod of 14/10-hour light-dark cycle. Sodium chloride (NaCl) solution of 200 mM concentration was added into the nutrient solution at three leaf stage of cotton plants. Root and leaf samples were collected at 0, 1, 3, 6 and 12 hours after salt stress. All samples were immediately frozen in liquid nitrogen and stored at -80 °C for RNA extraction.

### RT-qPCR and RNA sequence

The RNA expression data of 64 genes according to salt stress and control environments in 0, 1, 3, 6 and 12 h time intervals were obtained from cotton functional genomic database (cottonFGD) (https://cottonfgd.org). The reads per kilobase of exon per million reads mapped (FPKM) expression values of genes was altered into log10 values for the construction of heat map. The RNA from root and leaf samples was extracted using SIGMA Life Science RNA kit protocol (sigma-aldrich.com). The concentration and quality of extracted RNA samples were measured in NanoDrop spectrophotometer (2000). The RNA samples were selected based on the standard concentration at 260 to 280 and the quality range from 1.85 to 2.0 for the next step. Trans Gen Biotech kit was used for the synthesis of cDNA. National Centre for Biotechnology Information (NCBI) website was used to design primers of 12 highly upregulated genes. Further information about primers is given in S1 Table. The RT-qPCR was done using a 7500 PCR system. A total of 20 μl reaction volume was maintained, which included SYBR green (10 μl), forward/reverse primer (2 μl), distilled water (6 μl) and Ghactin7 (2 μl). For each sample, three replications were performed for RT-qPCR. Expression values of genes were calculated with the help of following formula E = ^2-ΔΔCt^.

## Results

### Segregation distortion (SD) pattern analysis

According to Chen et al. [17], a genetic map entailed of 2922 markers amplifying 2763 loci were distributed into 26 linkage groups corresponding to 26 chromosomes [17]. The 384 markers out of 2763 were distorted, accounting for 0.14% of markers on 18 chromosomes. The 29 SDRs were observed on Chr01, Chr04, Chr05, Chr06, Chr07, Chr08, Chr10, Chr12, Chr13, Chr15, Chr16 Chr17, Chr19, Chr21, Chr22, Chr23, Chr24, and 26, each one of them possessing a different SDRs, nominated as SDR1-1, SDR2-15, SDR3-17, SDR4-4, SDR5-22, SDR6-22, SDR7-22, SDR8-22, SDR9-5, SDR10-19, SDR11-19, SDR12-6, SDR13-6, SDR14-07, SDR15-16, SDR16-16, SDR17-08, SDR18-24, SDR19-24, SDR20-23, SDR21-23, SDR22-10, SDR24-21, SDR25-12, SDR26-12, SDR27-26, SDR28-26, and SDR29-13, respectively (Fig 1). The distorted markers were observed to be unevenly dispersed throughout the genome. All loci in SDR3-17 on D3 (Chr.17) deviated towards the male parent *G*. *darwinii*, while 90% of the loci in 4 SDRs on D4 (Chr.22) diverged towards the recurrent parent *G*. *hirsutum* CCRI12.

**Fig 1:** (A) Collinearity between a genetic and physical map of At and Dt subgenome of *G*. *hirsutum*. (B) Collinearity Analysis between genetic map and physical map of GbAt and GbDt of *G*. *barbadense*. Different colors indicate the several syntenic blocks on chromosomes.

Similarly, all loci in SDR20 to 23 were twisted towards the heterozygote, whereas the entire loci in SDR21 to 23 diverged towards their recurrent parent. Out of 29 identified SDRs, 8 were positioned on At subgenome and 21 were present on Dt subgenome. Various groups of SD sites were detected on Chr16, Chr22, and Chr23. The highest segregated distorted loci were observed on Chr22 with 64.28%, followed by Chr16 with 55.55%, while minimum segregated distorted loci were noted on Chr21 and Chr07 with 5.26% and 4.56%, respectively [17]. Certain regions on the chromosomes had longer clusters of SD sites and the name of these regions were known as SDRs as shown in Fig 1 and S1 Table, and Table 1.

**Table 1:** Detail of SDR markers on different chromosomes of cotton.

Chromosome	Number of SDR regions	Number of markers in SDR regions	Total number of markers	Percentage of SDR markers (%)
Chr-1	1	12	100	0.12
Chr-4	1	06	49	0.12
Chr-5	1	15	160	0.09
Chr-6	2	34	84	0.40
Chr-7	1	05	105	0.05
Chr-8	1	19	110	0.17
Chr-10	1	07	83	0.08
Chr-12	2	16	112	0.14
Chr-13	1	06	100	0.06
Chr-15	1	12	119	0.10
Chr-16	2	50	90	0.56
Chr-17	1	09	87	0.10
Chr-19	2	42	163	0.26
Chr-21	1	05	95	0.05
Chr-22	4	63	95	0.66
Chr-23	2	41	95	0.43
Chr-24	2	12	127	0.09
Chr-26	2	30	126	0.24

### Collinearity analysis of the genetic and physical map of *G*. *hirsutum*

Collinearity analysis was done between constructed genetic maps with reference to *G*. *hirsutum* genome. A total 384 SSR markers were blasted in At and Dt subgenome of *G*. *hirsutum* obtained from SDRs. After elimination of redundant markers, 55.46% of mapped markers showed consistency between two maps with 62 markers found similar with At, while 151 markers with Dt subgenome. The 171 markers were not similar with a physical map of the reference genome (Fig 1A). For collinearity analysis, 213 markers positions were analyzed for comparison between physical and genetic map of Dt (151) and At (62) sub-genome of upland cotton. The At sub-genome sequences showed linear similarity in sequences from 1 to 13 such as chr4 showed similarity with A4 and chr5 with A5 in At sub-genome. While in the Dt sub-genome, random collinearity among chromosomes has been observed for example chr4 showed similarity with D22 and chr5 with D19. Most of the markers have good collinearity blocks. However, all chromosomes showed good syntenic blocks with Dt subgenome and At subgenome. (Fig 1A and S2 Table). Comparison analysis of physical and genetic maps from the sequences of markers is important in confirming the order of genetic markers [39].

### Collinearity between genetic map and physical map of (GbAt) and (GbDt) sub-genomes of *G*. *barbadense*

The 384 SSR markers were obtained from SDRs of genetic map blasted in two sub-genomes of *G*. *barbadense*. From all markers in GbAt (120) and GbDt (228), 62 and 147 markers were aligned to assembled genome of *G*. *barbadense* (GbAt and GbDt, respectively). In GbAt (51.66%) and GbDt (64.47%) of markers in *G*. *barbadense* presented similarity between the physical and genetic map. Nevertheless, 54.42% of SDRs markers were in non-conformity between the two maps. Collinearity results indicated that GbDt genetic map was more closely related to the physical map and the maximum number of markers showed similarity in GbDt as compared to GbAt. However, decent syntenic blocks were noted between genetic map chromosomes and sub-genomes of *G*. *barbadense* (Fig 1B and S3 Table). The arrangement of homology between chromosomes indicated that some genes may be transferred into the population from wild parent. Previous reports suggested that the rate of gene introgression from *G*. *darwinii* into *G*. *hirsutum* was higher than *G*. *barbadense* into *G*. *hirsutum*. The 43.7% of introgression has been reported from wild species as compared to other local accessions, which was 18.4%. Interestingly, the rate of gene introgressions from the wild and developed accessions into *G*. *barbadense* was 33.1% and 27.1%, respectively. Therefore, the flow of genes from wild species into *G*. *hirsutum* was higher as compared to *G*. *barbadense* [40].

### Identification of genes and phylogenetic analysis

In order to determine the genes in segregation distortion loci (SDL), sequences comprising SSRs were retrieved from CottonFGD. The physical locations of the SDLs were recognized by using the sequences of SSR markers as a query in BLASTx against the reference genome (TM-1) [41]. The genes in the adjacent region were obtained for every SDL using physical position and cotton genome database. We obtained 214 SDR marker sequences from AD genome out of 384 sequences. We conducted a BLAST search and mined 568 genes in three cotton species, including *G*. *hirsutum* (284), *G*. *arboreum* (142) and *G*. *raimondii* (142) within the 29 SDR regions of 18 different chromosomes. We further grouped 568 genes according to their respective domains. The 23 uncharacterized genes were found in addition to three gene families, which were then subjected to phylogenetic analysis to investigate the evolutionary association among uncharacterized genes. It is believed that these are deliberated to be highly conserved and have a key role in plant biology [31]. Three top domains, including zinc finger (PF01754), Pkinase (PF00069) and MYB (PF00249) domains, are known to play a vital role under biotic and abiotic stress conditions. Seventy-one genes belonged to the zinc finger family, 18 to the Pkinase domain and 16 to MYB domain, while among 23 uncharacterized genes, 15 remained uncharacterized with no known function. Whereas, eight genes were present in PLATZ transcription factor family of proteins (S4 Table), found in 94 species with a total of 1374 sequences, containing the following InterPro domains (Fig 2). PLATZ1 protein in the peas is known as zinc-dependent DNA-binding protein involved in the transcriptional repression of A/T-rich sequences.[42]. All the gene sequences were used in MEGA (v6.06) software to develop a phylogenetic tree using the neighbor-joining method, with 1000 bootstrap replicates. The reliability of the phylogenetic tree was also confirmed by minimum evolution method. Both methods employed resulted in the creation of identical gene trees, implying that both methods are consistent with each other. The phylogenetic tree consisted of 128 genes (S4 Table). The total number of genes in the three cotton species were; *G*. *hirsutum* (64), *G*. *arboreum* (32) and *G*. *raimondii* (32) (Fig 2). The PF00069 belonging to the superfamily Pkinase was used as a reference because 8 out of 23 uncharacterized genes were cultured with this protein domain. From the previous reports, protein kinases are known to regulate the response of plants against water and salt stress [43]. The remaining 15 genes were more closely related to zinc finger domain. It is hypothesized that since these genes closely cluster with known stress-responsive genes playing crucial roles in plant survival, they can be predicted to have the same function assigned to proteins based on bioinformatic tools in comparative genomics as performed below [44]. Furthermore, eight uncharacterized genes in *G*. *hirsutum*, *G*. *arboreum* and *G*. *raimondii* indicated as *Gh_D09G1346*, *Gh_A09G1344*, *Gh_D04G1032*, *Gh_A04G0577*, *Ga04G0907*, *Ga09G1638*, *Gorai*.*009G411100* and *Gorai*.*006G159900*, grouped close to *Ga09G2796* and *GhA09G2172*, which has the known function of a protein related to Pkinase domain. The *GhA04G0577* gene, for instance, has a homolog in Arabidopsis At3g50808, grouped close to the Pkinase of *G*. *arboreum* and *G*. *raimondii*. This indicates that this gene may flow from *G*. *arboreum* and *G*. *raimondii* to *G*. *hirsutum* in equal proportions. Similarly, *Gh_A12G0242*, *Gh_D12G0241*, *Gh_D04G1604* and *Gh_D04G1606*, *Gh_A03G1703*, *Gh_A03G1703*, *Gh_D02G2124*, *Gh_A13G0319*, *Gh_D13G0358*, *Ga14G0186*, *Ga13G0339*, *Ga03G2503*, *Gorai*.*008G027200*, *Gorai*.*012G151300*, *Gorai*.*005G241600* and *Gorai*.*013G039300* were closely grouped to *Gh_A10G1525*. The *Gh_A10G1525* is a well-known zinc finger protein that alters the reaction of plants under osmotic and salt stresses [45]. Most of these excavated genes, particularly uncharacterized ones, belonged to the single protein domain, which means that these genes were greatly conserved. Three families were clustered into distinct groups in the phylogenetic tree with each family illustrated by a different color as presented in Fig 3. These genes were distributed on 24 chromosomes. Furthermore, a comparative analysis was done to identify the orthologous gene pair among the Pkinase, zinc finger and MYB gene families between upland cotton, *G*. *arboreum* and *G*. *raimondii*. All genes in functional groups present in At subgenome of *G*. *hirsutum* paired with its orthologs in the A genome of *G*. *arboreum*, while those in Dt subgenome had their orthologs in D genome of *G*. *raimondii*. The occurrence of these ortholog genes in the related cotton genomes further affirms the evolution of tetraploid cotton, *G*. *hirsutum*, which supposedly arose as a result of an entire genome duplication event between the D and A subgenomes [46].

**Fig 2:** (A) Designates an entire number of cotton genes in zinc finger Pkinase and MYB and (B) total genes in individual subfamilies.

**Fig 3:** Phylogenetic tree relationship of three gene families with uncharacterized genes in *G*. *hirsutum*. Dissimilar border line depicts various gene subfamilies.

In *G*. *hirsutum*, maximum number of genes (5) was present on chromosome At09, At12, Dt04, Dt08 and Dt09, while minimum (1) was found on At06, At07, Dt06, Dt07 and Dt13. Similarly, the highest genes were detected on chromosome A09 in *G*. *arboreum* and D06 and D12 in *G*. *raimondii*, respectively, while the lowest density was detected on chromosomes A06, A07, D01, D10 and D13 with just a single gene per chromosome (S2 Fig).

### Structure analysis and physiochemical properties of the stress-related gene families with uncharacterized genes obtained within the SDRs

Structure analysis of genes gave shreds of evidence to support the phylogeny within a gene family [47]. Gene structural diversity provides conceivable indications about the mechanisms of evolution of new multigene families [48]. To gain further insight, an exon/intron organization in the full-length cDNAs with their corresponding genomic DNA sequences of individual genes in upland cotton was analyzed.

Gene Structure Display Server (GSDS v2.0) was used to illustrate gene structures displaying the relative positions of exons and introns in three gene families with uncharacterized genes; (Fig 4A and S5 Table). About half (49.21%; 31) of the total genes (63) had no introns, while the other half (50.79%, 32) contained introns which varied from one to eight. Moreover, among intron-containing genes, nine had a similar structure containing either six or eight introns, while the rest were disrupted by only two or three introns. The highest exons and introns were observed in *Gh_A06G1427*, *Gh_D06G1775*, *Gh_A10G2148* and *Gh_D10G2395* (nine exons, eight introns), while minimum number were two exons and one intron in most of the genes. Interestingly, we found that 31 genes had only one exon and no introns in their sequences. A higher degree of exon-intron match was observed for the genes clustered together. The exon/intron structure of genes was constant in the results of a phylogenetic tree. Significant structural diversity indicates the different functions of these genes.

**Fig 4:** (A) *G*. *hirsutum* genes structure demonstrated by GSDS 2.0. Exons and introns are depicted with blue and red lines. (B) Different cellular compartments indicate the genes localization.

Physicochemical parameters of three cotton families with uncharacterized genes were measured using the online tool, ExPASy [49]. The physiochemical properties of these genes showed significant variations. The grand average of hydropathy (GRAVY) gained from ExPASy designated that all of the identified proteins were hydrophobic, having GRAVY values < 0, these results are consistent with those of the Pkinase and zinc finger proteins in cotton and *Arabidopsis thaliana* [50]. All genes in *G*. *hirsutum* had negative GRAVY values ranging from -1.527 (*Gh_D09G0631*) to -0.051 (*Gh_D12G1454*), which implied that cotton zinc finger, Pkinase, MYB and uncharacterized genes are hydrophobic in nature. These properties mostly occur in stress-related genes, for instance, late embryogenesis abundant (LEA) genes have less than zero GRAVY value [51]. The physiochemical properties of these genes showed significant variations in protein lengths, in case of *G*. *hirsutum*, ranged from 75 aa (*Gh_A12G1443*) to 672 aa amino acids (*Gh_D12G1454*). The molecular weight vary from 8.579 kDa (*Gh_A12G1443*) to 75.042 kDa (*Gh_D12G1454*) and isoelectric point ranged between 3.919 (*Gh_D01G0589*) and 10.71 (*Gh_D09G0671*). High net charge and lower GRAVY values have been previously noted for these families and has been a distinctive feature of Pkinase genes in cotton and Arabidopsis [52]. Many stress-inducing proteins are usually characterized by low hydrophobic rates and higher charge, this function gives zinc fingers, Pkinase, MYB and uncharacterized genes to form a stretchy three-dimensional molecular structures, for instance, molecular chaperones, which enable the plants to resist drought [53]. Furthermore, hydrophobic proteins are arranged in such a way that nonpolar amino acids are buried inside the core of the protein, shielded from the solvent. This feature is commonly present among transmembrane proteins such as aquaporin’s (AQPs) and water channel proteins. It plays a critical functional role in enhancing the tolerance of plants against salt and water stresses [54].

The online WoLF PSORT analysis indicated that genes were distributed into six sites. Most of the genes were confined to nucleus (42) and chloroplast (14), accounting for 65.62% and 21.87% of all three cotton families and uncharacterized genes, respectively. Whereas, a lesser number of genes were observed in plasma membrane (3) vacuole (2), mitochondria (1) and extracellular matrix (2) (Fig 4B and S6 Table).

### Gene annotation by GO analysis

We conducted a BLAST search and mined 284 genes of *G*. *hirsutum* within 29 SDRs of 18 different chromosomes. These genes were distributed on all 26 chromosomes. The dominant domains contained 52 genes of the top three salt-tolerant gene families and 12 uncharacterized genes were present on all 24 chromosomes. The highest number of genes were present on the chromosomes chr09 (5) and chr12 (5), while the least number were found on chr06 (1) and chr07 (1). Gene Ontology analysis has been classified into three categories; such as molecular functions (MF), cellular components (CCs) and biological processes (BP) [55]. Putative functions of 64 genes were predicted using the cotton functional genomics database (https://cottonfgd.org). In biological processes, the functions include phosphorylation (34%), phosphate metabolic process (33%) and phosphorus metabolic process (33%). The molecular function of genes can be outlined as kinase activity (8%), DNA binding (14%), zinc ion binding (10%), transition and metal ion binding (10%), binding (29%), protein tyrosine kinase activity (29%), nucleic acid binding (14%), and transferase activity, transferring phosphorus-containing group (8%) (Fig 5).

**Fig 5:** The 64 genes of *G*. *hirsutum* were classified into biological processes and molecular functions.

### Duplication and syntenic analysis of genes

The expansion of gene families has been known to have occurred by three processes such as whole genome, segmental and tandem duplications [56]. To outline these, genomes of three cotton species were gathered for checking the associations between the gene synteny and duplication in three gene families with uncharacterized genes.

MCScanX software was used to determine the duplication events and Circos for the visualization of data. Results showed the duplication of 89 genes across the tested cotton species (Fig 6 and S7 Table). The presence of more than two genes on same chromosome in tandem is known as tandem duplication, while duplication of a gene on different chromosomes is known as segmental duplication [57]. In the current study, cotton genes construct groups that possibly explain the process beyond their evolution. Maximum gene duplication occurred between *G*. *hirsutum* and its progenitors, *G*. *raimondii* and *G*. *arboreum*, implying that polyploid AD genome had arisen as a result of duplication between A and D genomes leading to the development of novel species in *G*. *hirsutum*. Most of the genes showed segmental duplication, suggesting that this was a major reason for the origination of different genes families (Fig 6). Furthermore, we calculated the nonsynonymous (Ka), synonymous (Ks) and Ka/Ks values for the homologous gene pairs in *G*. *hirsutum* to further reveal the mechanism of gene deviation after polyploidization. The Ka/Ks values are indicative of the selection pressure acting on protein-coding genes and can be used as an index to conclude the magnitude of selective constraint and positive selection. It has been reported that there is a systematic bias in the process of nucleotides substitutions in some species. Variations in the composition of an amino acid are greater due to species diversity and higher rate of mutations [58, 59]. Generally, Ka/Ks value >1 indicate positive or favorable selection due to profitable mutation effects. A Ka/Ks ratio of 1 represents a neutral selection, while the Ka/Ks ratio <1 indicates negative selection or harmful mutation effects, also known as purifying selection [60, 61]. The Ka/Ks value of ortholog genes showed that 76 gene pairs have <1 value, while 17 gene pairs have >1 Ka/Ks values, indicating that all genes have gone through positive and purifying selection at the evolution time (S8 Table). In a previous study, Magwanga et al. [28] found that Ka/Ks value <1 for 156 paralogous pairs and >1 for 20 pairs of LEA gene family in cotton. The maximum Ka ratio of 0.0469 was recorded for gene pairs in Dt vs DD genome of gene pairs. While the Ka value of At vs AA extended between 0–0.0145. As shown in the Fig 6A and S8 Table, Ka/Ks value was greater for AA vs DD genome pair (2.872) as compared to Dt vs DD and At vs AA. These findings are related to earlier studies with other identified gene families (i.e., in ROS gene family Ka/Ks value was detected 1.0 for AA vs DD, 1.8 for Dt vs DD and 1.7 for At vs AA genomes) [62].

**Fig 6:** (A) Circulation of Ks ratios among orthologous gene of diploid genomes (A & D) and *G*. *hirsutum* (Dt & At). (B) Determination of Ka/Ks value between the two diploid genomes (A & D) and *G*. *hirsutum* (Dt & At). (C) Syntenic relationships among all homologous genes *G*. *hirsutum*, *G*. *raimondii* and *G*. *arboreum*. Every chromosome in the particular subgenome is indicated with a similar color.

Synteny analysis showed a total of 27, 32 and 30 orthologous syntenic blocks between At and A, Dt and D and A and D, respectively (Fig 6C). It is interesting to note that more genes were observed between the syntenic blocks among the three cotton species, for instance, at most, four genes were found within the syntenic regions between At and A on chromosome 09 and 12. However, at most, 5 genes were found between Dt and D (Dt12 and Dt09). Similarly, a maximum number of four genes have been found on A09 and A12 within the syntenic regions between A and D. The higher number of stress-related genes detected within the equivalent syntenic regions showed that these regions have been highly conserved indicating their integral role within the plants. These results support the principle of asymmetric selection of genes within the genomes [63].

### Cis-elements analysis

We have examined the three major subfamilies and uncharacterized genes to determine if there could be any known regulatory elements which can play their roles in various biotic and abiotic stress conditions [64]. In the promoter regions, cis-acting elements act as the molecular switches to regulate the stress-responsive genes by providing binding sites to the transcription factors. Upstream 1.5 kb genomic sequences of each gene relative to TSS (translation start site) were collected to examine the regulatory interactions between transcription factors and promoter elements. Results showed that these genes had diverse functions because of the presence of different types of cis-elements in their promoter regions. In the analysis, all genes were related to either abiotic or biotic stress-responsive cis-regulatory elements. Hence, several cis-elements that play regulatory role in plant stress were identified, including MYBS (abiotic stress tolerance), Box 4 (light responsiveness), TGA-element (auxin-responsive element) and ABRE (salt, drought and abscisic acid responsiveness) (Fig 7, S9 Table). Promoter region analysis of all genes has shown the presence of various stress-responsive cis-acting regulatory elements, i.e., DRE, that acts as activators of various genes expressed under drought, salinity and cold stresses; ABRE (CGCACGTGTC), which functions in the early response to the stress conditions and MYB (CAACTG), which is induced by mechanical stresses and abiotic stresses such as wounding or elicitor treatment among others. Likewise, TCA-elements and TGACG-motif are responsive to methyl jasmonate (MeJA) and salicylic acid (SA) treatments [65]. These elements, particularly the ABREs and CAAT-box, were found abundantly in the *G*. *hirsutum* genes, which indicate their possible role under salt stress conditions. While, the other identified cis-regulatory elements i.e. ABRE, NAC and MYB are already known to be associated with the top-ranked plant stress-responsive genes [66]. The recognition of these main cis-elements in the promoter region of 64 candidate genes indicated that they are directly involved in salt stress mechanisms, accordingly which might help in resolving the salt stress pandemics in cotton. MYB are the main cis-acting promoter elements that play an important role in the ABA-dependent signaling pathway under various abiotic stresses [66]. Similar findings, with the identification of stress-responsive cis-elements, have been reported for many genes in tomato [67], Arabidopsis [68], Chinese plum and cotton [59].

**Fig 7:** Cis-element of genes that responded to salt stress.

### miRNA target analysis of genes

The function of genes is controlled by numerous biomolecules, in which miRNA had been found to play a basic part by controlling the gene expression levels [69]. A rising indication proposed [48] that miRNA plays a significant role in plants under stress conditions by targeting the gene expression levels [70]. In cotton, a group of miRNAs and their target genes are reported to respond under salt and drought stresses [71]. In order to check whether any of the 64 *G*. *hirsutum* genes have been targeted by any known ghr-miRNAs, we analyzed the putative target sites of cotton miRNAs in CDS sequences using the psRNATarget server. A total 39 genes out of the 64 were found to be targeted by 234 ghr-miRNAs, including its types based on different origins, translating to 60.93% of all the genes (S8 Table). The highest levels of target were detected on the following genes including *Gh_A05G2890* and *Gh_D06G1775*, each have 19 ghr-miRNAs.

The highest level of miRNA target was noted for ghr-n58, found to target 14 genes and ghr-mirR530a, ghr-mirR530c, ghr-mirR156e and ghr-mirR418, each targeted 12 genes as described in S10 Table. The miRNAs targets were observed to be very high, with a single gene being targeted by a minimum of one to a maximum of 14 miRNAs. For instance, ghr-mirR156e targeted 12 genes involved in salinity and drought stress [71]. Twenty-two zinc finger genes were targeted by 14 miRNAs, and nine genes of Pkinase were targeted by five miRNAs and eight uncharacterized genes were the targets of five miRNAs, while no MYB genes were found to be targeted by any of the miRNAs. The ghr-miR482 was found to target the uncharacterized genes *Gh_A09G1344* and *Gh_D09G1346*, as well as *Gh_D09G1323* and *Gh_D06G1775*; which belongs to zinc finger and Pkinase gene domains, respectively. Similarly, different variants of ghr-miR2949 targeted the uncharacterized genes *Gh_D02G2124*, *Gh_A03G1703*, and *Gh_D10G2395*, *Gh_A10G2148*, both of which belongs to the Pkinase domain. These results are in conformity with the phylogenetic analysis in which the uncharacterized genes clustered with the Pkinase and zinc finger gene families. Therefore, cementing the probability that these genes are most likely involved in the stress response mechanism. The high miRNA targets detected for these genes showed that the genes obtained from the 29 SDRs on 18 chromosomes have a significant role in various biological processes within the plant. The high number of miRNAs targeting the genes could possibly be correlated directly or indirectly with their tolerance levels to abiotic stresses, especially salinity.

The miRNA/sRNAs mediated post-transcriptional processing have been linked to act in response to salinity and water deficit conditions [51]. Therefore, our results showed that these miRNAs have a role in the regulation of SDR genes against abiotic stress.

### RNA sequence data of salt tolerant genes

RNA sequence of an organism is an important tool that reveals the genetic role of genes. It provides information about the expression levels of genes under various biotic and abiotic conditions as well as their abundance in different plant organs. In this study, RNA sequence data for the genes at the SDRs were obtained at 1, 3, 6 and 12 hours of control and salt stress conditions. In this context, data of 64 salt responsive genes at the identified SDRs were downloaded from cotton functional genomic database (cottonFGD). Sequence data of 64 salt-responsive genes was changed into log10 and used to determine the expression levels under control conditions and various time intervals (1, 3, 6 and 12 hours) of salt stress. These 64 salt responsive genes were divided into three different groups. In group 1, most of the genes were upregulated, in group 2 genes exhibited differential expression, some of them showed upregulation, while others showed down-regulation and even no expression, and in the group 3; most of the genes were upregulated and showed partial expression and even no expression (Fig 8A). The 41 genes were up-regulated out of 43 and 19 were down-regulated out of 21, in control and stress environment. These 41 (61%) genes were up-regulated in both stress and control conditions, while only 19 (29.7%) genes were found to be commonly down-regulated in control and stress environments (Fig 8B). Fifteen genes from the first group were highly up-regulated under control and salt stress environment. These highly up-regulated genes including *Gh_A01G1773*, *Gh_D01G2015*, *Gh_D04G0980*, *Gh_A04G0524*, *Gh_A05G0679*, *Gh_A12G2033*, *Gh_D12G2211*, *Gh_D04G0444*, *Gh_D09G0146*, *Gh_A09G0154*, *Gh_A10G1525*, *Gh_D10G1776*, *Gh_A05G2890*, *Gh_D09G2382* and *Gh_A09G2172* were selected for further validation.

**Fig 8:** (A) Expression patterns of 64 SDR genes in relation to salt stress. Red lines indicate up-regulated genes and blue color indicates down-regulated genes, while the white line shows no expression of genes. (B) Diagram representing the upregulated and down regulated genes in control and salt stress conditions.

### Gene’s validation under salt stress

In response to any biotic and abiotic stress conditions, plants have to adjust their transcriptomic profile according to the environment [72]. Expression levels of responsive genes help us to know the role they may play under stress. For RT-qPCR analysis, we selected the fifteen highly up-regulated genes according to the RNA sequence data (S1 Table). Roots and leaf samples were used to check the gene expression levels at different time intervals under stress conditions. For the RT-qPCR analysis, wild *G*. *darwinii* and *G*. *hirsutum* species were cultivated under controlled conditions. Expression profiles of selected genes were checked by RT-qPCR from the root and leaves samples at 0, 1, 3, 6, and 12 h after salt treatment. The results depicted in Fig 9 show that in 200 mM salt treatment, genes depicted differential expression in roots and leaves.

**Fig 9:** (A) RT-qPCR expression profiles of 12 *G*.*hirsutum* genes. *G*. *darwinii* (Gd) and *G*. *hirsutum* (Gh). Red blocks indicate up-regulated and blue shows down-regulated genes however white blocks show zero expression. (B). Common up-regulated genes in leaf and root tissues of *G*. *darwinii* (Gd) and *G*.*hirsutum* (Gh).

In *G*. *hirsutum* and *G*. *darwinii*, expressions of genes were the same as in RNA profile and formed two clusters. Group 1 had four genes, which were up-regulated in different tissues of *G*. *darwinii*. All of the genes were upregulated in leaves, while roots of *G*. *hirsutum* showed down-regulation of genes at 1, 3, 6, and 12 hours after salt treatment, excluding *Gh_A04G0524*, which showed a lower expression. The second group had 11 genes, in which most of the genes were depicted to have a different expression, only one gene *Gh_D10G1776* was expressed in leaves of *G*. *darwinii*; while six genes were down-regulated in the roots of *G*. *hirsutum* (Fig 9A). *Gh_D04G0980*, *Gh_A04G0524* were highly upregulated in root tissues of the two species after 12 hours of exposure to salt stress, showing their salt-resistant role in root development. The *Gh_D01G2015* was highly upregulated in the leaves of parental species. Moreover, *Gh_D01G2015* and *Gh_A01G1773* had a higher expression in *G*. *darwinii*, while the opposite expression was observed in *G*. *hirsutum*. The two genes are narrowly connected to the SSR markers HAU3297 and HAU1012 on Dt and At genomes, respectively. The two markers are observed to be novel markers associated with potential stress-responsive genes.

The details of the identified genes closely linked to markers are shown in S3 Fig. These two candidate genes in *G*. *darwinii* showed high expression in root tissue after 12 hours of salt stress. Their role was depicted in the development of root systems for improving salt tolerance. A maximum number of eight genes, approximately 53.3% of all genes, were simultaneously upregulated in leaves and roots of *G*. *darwinii* and leaves of *G*. *hirsutum*, whereas only four genes (26.75%) were commonly upregulated in leaves and roots of both cotton species (Fig 9B). These results showed that few key alleles from wild tolerant species may have transferred into developed F_2_ populations, which can help as a background to overcome salt stress effects on cotton plants. Maximum genes showed higher levels of expression in the roots of *G*.*darwinii*. This is understandable because of the fact that the first and main response against salt stress is initiated in the roots of plants. Few genes were highly upregulated in leaves of *G*. *hirsutum*. Most of the genes were present in *G*.*darwinii* than the *G*. *hirsutum*, suggesting that wild species were more salt-stressed as compared to *G*. *hirsutum*. The higher expression of FBA and Pkinase genes were previously observed in *G*. *darwinii* and was found to be lower in *G*. *hirsutum* [73].

## Discussion

Segregation distortion (SD) is an anomaly of estimated frequencies from the Mendelian ratio in a segregating population [74]. The SDRs have been noted in both intra and interspecific crosses and are one of the main causes for the evolution of new species [17]. Segregation distorted markers have been previously reported in numerous plants including maize, [4], barley [5], potatoes [6], wheat [7], rapeseed [8] and cotton [9]. The main effect of SDRs has been reported in breeding applications and gene mapping; however, this is a commonly found trait in plants. The study of SD is significant because distorted markers could be linked to important genes, and these genes may be beneficial or lethal to the organism. Therefore, it is important to include the segregation distortion markers since the exclusion of such markers could bias the data and result in the loss of some important genetic information.

We noticed 29 SDRs on 18 chromosomes from a genetic map. The percentage of segregation distortion presented in the map used in this study was 13.18%. The largest SDRs were observed on chromosomes 16, 19 and 22. Previously published genetic maps in cotton revealed that a higher number of SDRs were situated on chromosomes 02, 16 and 18 [60]. Similarly, Kirungu et al. [16] observed the highest segregation distorted markers on chromosomes 02 and 07 in the genetic map of two wild cotton species., Chromosome 02 had the least mapped markers but had the highest percentage of segregation distortion, ranging between 42.8% and 76.08% [16]. Entire loci in SDR3-17 (Chr.17) and SDR20-23 (Chr23) diverged to *G*. *darwinii*, while 90% of the loci in four SDRs on D4 (Chr.22) and SDR21-23 (Chr23) deviated towards the female parent *G*. *hirsutum* CCRI12. sBased on our results, we determined that SDRs on chromosomes might also contain some important genes. These SDRs might have arisen as a result of pre-or post-zygotic selection and chromosome loss/rearrangements. Therefore, it is necessary to excavate genes in these regions. Key genes will help solve the problem of SDRs by genome-wide association studies (GWAS) and determination of main characters e.g. Bovill et al. [76] recognized the crown rot resistance gene in SDR of the wheat crop; correspondingly, Sr36 gene was noticed on chromosome 2 B in SDR [75, 76].

Cotton production has been decreased due to major effects of abiotic and environmental stresses as well as the narrow genetic base of best cotton varieties [77]. To solve these problems, it is necessary to transfer the agronomic characters of wild progenitors into cultivated cotton. The wild cotton progenitors are important for alleviating different biotic stresses and abiotic epidemics in plants [18]. Under the constraints of an unpredictable weather patterns; including low precipitation, high temperatures and increased salinization of cultivable lands, the plants have opted to evolve multiple complex regulatory mechanisms to detect and generate signals modulating the expression of numerous plant transcription factors (TFs) with diverse roles in stress tolerance. Therefore, the detection of the 128 myriad genes of the top three salt-tolerant gene families with uncharacterized genes based on already developed highly dense genetic map in cotton, could offer a better alternative in solving the problem of salt stress, in cotton breeding approaches.

From the phylogenetic analysis, 128 genes were categorized into three subfamilies such as zinc finger, MYB and Pkinase playing key functional roles in abiotic stress resistance and characterized the potential function of 23 uncharacterized genes. Identified genes in *G*. *hirsutum* were doubled as compared to *G*. *arboreum* and *G*. *raimondii*, indicating that whole-genome duplication (WGD) was a major reason for the extension of these gene families [78]. *G*. *hirsutum* species was originated from the progenitors of *G*. *arboreum* and *G*. *raimondii* during duplication and polyploidization processes [79]. Evolutionary analysis has signified that most of the angiosperms have gone through one or multiple polyploidization events in their evolutionary histories [80, 81]. Similar distribution of genes have been noted in CDK *G*. *hirsutum* (31), *G*. *arboreum* (15) and *G*. *raimondii* (12) genes and as well as in FBA *G*. *hirsutum* (19); *G*. *raimondii* (9) and *G*. *arboreum* (9) genes, respectively [82]. These results indicate an important role played by these group of genes in plant growth and developmental processes [68].

Generally, gene duplication incident is considered to be a key driving force for exploring new biological functions, evolutionary implications and expansion of gene families [83]. Therefore, cotton being typically allotetraploid is a model crop to study evolution and polyploid formation [79]. Expansion of gene family has been evolved by segmental, tandem, and whole-genome duplication processes [56]. Good collinearity blocks were observed in orthologous genes between two subgenomes of *G*. *hirsutum* in the same way as the A and D genomes as shown in Fig 6. In order to estimate evolutionary patterns, such as the extent of selection pressure by calculating synonymous/non-synonymous substitution ratios (Ka/Ks); imparted useful information about positive, purifying and neutral selection of gene pairs divulging the rate of divergence [40].

An increase or decrease in exons or introns can be attributed to integrations and realignments of gene fragments. Consequently, structural variations in genes played the main role in the origination of new families [56]. The current study illustrates such diversification process in the form of genes having very similar structures, with exactly half (31) of the genes not disrupted by introns, with a single exon and no introns. Our outcomes are similar to earlier results, 45 percent of Arabidopsis and 41 percent of *Oryza sativa* have intron less F-box genes. In *O*. *sativa* (19.9%) and Arabidopsis (20.7%) intron-less genes were prevalent in the entire genomes [68, 69]. It has been assumed that intron-containing gene would miss various introns instantaneously by retro-transposition, giving rise to intron-less genes in the ancestors [84]. The intron-less genes are known to promote the efficiency of transcription initiation and elongation in spliced genes [85]. Introns affect the transcription process, meanwhile intron splicing needs a big complex of molecules, which takes a lot of time and effort for assembly and expression of these components [86, 87]. As a result, intron-less genes increase the initiation and elongation process of transcription than the gene splicing [85]. All of the identified proteins were found to be having GRAVY values lower than 0, lower GRAVY ratio indicated that these genes were hydrophobic in nature and most commonly present in stress- tolerant genes [88]. The similar gene structures and identical protein characteristics of similar subfamilies were consistent with the classification of a phylogenetic tree. Conversely, gene structure of different families have been dissimilar owing to different functions.

Gene ontology analysis classified the genes into a molecular function, biological process and cellular function. Based on GO annotation of SDRs, 64 genes of *G*. *hirsutum* were involved in molecular function and biological processes. In biological processes, numerous genes are linked with stress-related factors; for example, phosphorus metabolism method (GO:0006793) phosphate process (GO:0006796) and phosphorylation process (GO:00015210). Protein kinase play an important role in the signaling mechanism of plants under abiotic and biotic stresses [89]. Many genes were involved in molecular functions, i.e., transferring phosphorus group (GO:00017726), kinase function (GO:0016301), DNA ligation (GO:0004788), ribonucleic acid-binding (GO:0003677), zinc and metal ions binding (GO:0035803), RNA binding (GO:0005488) and tyrosine activity (GO:0004713) (Fig 6). *Gh_D09G2382* was associated with top-ranked Pkinase gene family with the six GO functions including ATP binding (GO:0004623), phosphorylation process (GO:0004143), diphosphate kinase process (GO:0005450), GATP biosynthesis procedure (GO:0005173), UTP biosynthetic activity (GO:0005127) and CTP synthesis process (GO:0005231); linked to the four uncharacterized genes, and have no GO functions. With the help of molecular functions, we understand the various approaches, a plant may adapt for its survival and tolerance against numerous stresses. The *Gh_D09G2382* gene GO functions indicates that it was involved in tyrosine kinase activity and abscisic acid signaling pathways [90]. Previous findings reported that Pkinase changed the reactions of plants in osmotic and salt stresses. *Gh_A10G1525* gene belongs to a zinc finger gene family, clustered with eight uncharacterized genes that have unknown functions. *Gh_A10G1525* was involved in DNA binding (GO:0003677). Zinc finger vigorously played a key role in the binding of DNA and RNA and protein recognitions [24]. The *Gh_A10G1525* is a well-known zinc finger protein that increases stress tolerance and plays a key role in plants against environmental stresses [45]. SDR genes demonstrated the significant role played by them in the evolution or synthesis of vital proteins with a profound function in improving tolerance levels of plants against numerous biotic and abiotic stresses.

The detailed study of MYB, Pkinase and zinc finger genes gained from SDR regions of the genetic map, cis-elements, miRNAs, and gene ontology suggested that these genes may play an important role in plant stress. Cis-elements are involved in the transcription process of genes which controls various hormone reactions and abiotic stresses. Hormones increase the adaptability of a plant in harsh conditions such as stress and fluctuating environments. ABRE, TCA elements, DRE, W Box and MBS were previously identified cis-elements related to plant hormones and abiotic stresses [91, 92]. Many **cis**-elements involved in stress mechanisms were abundantly found in three gene families of *G*. *hirsutum* and uncharacterized genes in SDRs, and MYB, demonstrating the key function of these cis-elements in salinity tolerance of *G*. *hirsutum*. 56 genes were regulated by MYB. MYB cis-element played a major role in the abscisic acid signaling pathway against salt, drought and cold stresses [66]. Similarly, ABRE is a vital cis-element and shows a significant function in abscisic acid signaling in reaction to various abiotic stresses [92]. An earlier study conducted in Arabidopsis described that cis-acting regulatory elements (CARE) increase tolerance in response to cold, salt and drought [93].

Current evidence demonstrated that miRNAs play a main function in biological and abiotic stress reactions in plants [94]. In *G*. *hirsutum*, an entire 64 genes were originated to be targeted by 234 ghr-miRNAs. The known miR156 targeted two genes (*Gh_A10G1525* and *Gh_D10G1776*) belonging to the zinc finger family, whose functions have been described. A recent study on miR156 primarily emphasizes its function in the regulation of flowering and morphological alteration. Evidence suggests that drought and salt stresses disturb the expression of miR156, representing its unique function under such stresses [71]. Another miRNA, miRNA482 regulates NBS—LRR protection genes in the course of fungal infection [95]. The four types of ghr-miR482 targeted three genes, i.e., ghr-miR482g targeted *Gh_D06G1775* and ghr-miR482c/f/i targeted two uncharacterized genes (*Gh_A09G1346* and *Gh_D09G1346*). Most of the targeted miRNAs were related to the stress tolerance and could play a functional role in response to NaCl stress and PEG stress [71]. miR399 maintained the structure of Arabidopsis by phosphate homeostasis mechanism after treatment of salt and drought [96]. Two types of ghr-mirR399g/h targeted *Gh_A04G0524* and *Gh_D04G0980* genes, which are the members of the zinc finger family. All genes are directly involved in defense and different stress mechanisms in plants.

Results of RT-qPCR, based on the heatmaps, revealed that 15 important genes have higher expression patterns in wild *G*. *darwinii* related to *G*. *hirsutum*. The best variety CCRI12 is more susceptible and wild *G*. *darwinii* shows tolerance in salt stress conditions. Moreover, two genes depicted highest expression levels in *G*. *darwinii*, *Gh_D01G2015* and *Gh_A01G1773*, while the same were down regulated in *G*. *hirsutum*. *Gh_D01G2015* and *Gh_A01G1773* belongs to zinc finger AN1 and A20 subfamily domains comprising of stress-related protein (Fig 8). The zinc finger subfamilies such as AN1 and A20 proteins were involved in physiological mechanism and help in enhancing the SAP in plants under dehydration, metals, salt and cold stresses [97, 98]. Zinc finger (C2H2) protein played a major role in physiological, growth processes and various environmental stresses in plants [99, 100]. The Arabidopsis ZHD protein is prompted using NaCl, abscisic acid, and PEG. The *OsSAP1* protein was firstly identified from A20-N1 plant, known to exhibit several stress tolerance reactions and found to be resistant against a cold, salt, and dehydration in genetically modified tobacco [101]. The *SbSAP14* gene in *Sorghum bicolor* is precisely prompted tolerance against oxidative stresses and took part in the antioxidant system of plants to enhance a salt stress tolerance [102]. Our findings confirmed that salt-tolerant genes have been introgressed from wild tolerant species. These results suggest that several of the candidate genes were salt-tolerant and can be helpful in the future for gene cloning, transformation, gene editing and development of resistant cotton varieties.

## Conclusion

Genetic map analysis played important role in the identification, gene mining, marker assisted selection and cloning. However, an in-depth analysis of SDR genes has not been yet studied. In this study, salt stress-related genes in segregation distortion regions of chromosomes were identified from genetic map of F_2_ generation in *G*. *hirsutum* CCR112-4/*G*.*darwinii*. Out of 384 markers, 214 marker sequences in segregation distortion regions of 18 chromosomes were used for further analysis. All markers had good collinearity in At and Dt subgenome of *G*. *hirsutum* and *G*. *barbadense*. In the F_2_ population, 128 genes of *G*. *hirsutum*, *G*.*arboreum* and *G*.*raimondii* were identified from SDR regions. A total of 128 genes were analyzed. Synteny analysis showed that the identified genes were extremely conserved, whereas duplication analysis signified that merely segmental duplication played a crucial function in the expansion of genes. In addition, phylogenetic analysis classified all genes into three major subfamilies and the uncharacterized genes clustered with either the protein kinases or zinc finger TF proteins. The gene structures showed that most of the genes were characterized with no introns. Additionally, we used RNA expression data to check the expression and function of genes against salt stresses. This study offers a detailed analysis of top three salt-tolerant gene families including Pkinase, zinc finger and MYB, besides it also helps in the identification of the function of uncharacterized genes found from SSR markers of SDR regions and expression levels of up-regulated genes in salt stresses. A further in-depth study of these families will support in understanding their roles in SDRs for future molecular breeding studies.

## Supporting information

S1 Fig Segregation distortion region (SDR) of 18 chromosomes in Map that have 29 SD regions. (DOCX)

S2 Fig Chromosomal distributions of zinc finger, Pkinase, MYB and uncharacterized genes on chromosomes of three cotton species. (DOCX)

S3 Fig Physical map presented the locations of the exact genes. NAU, HUA, DPL, BNL, TMD and others are the SSR markers, whereas Gh indicates the gene. Key genes are designated with red color.
(DOCX)

S1 Table PCR primers. (XLS)

S2 Table Assessment of collinearity of the genetic and physical map of Dt subgenome of *G*. *hirsutum*. (XLS)

S3 Table Collinearity analysis of genetic map to that of the physical map of (GbAt) and (GbDt) genomes of *G*. *barbadense*. (XLS)

S4 Table Protein kinase, zinc finger, MYB and uncharacterized genes identified in *G*. *hirsutum*, *G*. *arboreum* and *G*. *raimondii*. (XLS)

S5 Table The structural analysis of *G*. *hirsutum*. (XLS)

S6 Table Subcellular localization of genes. (XLS)

S7 Table Syntenic analysis of homologous genes among *G*. *hirsutum*, *G*. *arboreum* and *G*. *raimondii*. (XLS)

S8 Table Calculated, Ka, Ks and Ka/Ks ratio of orthologous pairs among three cotton species. (XLS)

S9 Table Cis-element of genes that responded to salt stress. (XLS)

S10 Table miRNA targets of genes. (XLS)
